The article "Time to First Sexual Experience and Its Determinants among Female Youths in Ethiopia: Survival Analysis Based on EDHS 2016" was published in 2022. Journal: Biomed Res Int.

# Time to First Sexual Experience and Its Determinants among Female Youths in Ethiopia: Survival Analysis Based on EDHS 2016

**DOI:** 10.1155/2022/5030902

**Published:** 2022-09-09

**Authors:** Tegene Atamenta Kitaw, Ribka Nigatu Haile

**Affiliations:** Department of Nursing, College of Health Science, Woldia University, Woldia, Ethiopia

## Abstract

**Background:**

The first sexual experience is the most significant event in a woman's life. Early sexual experience has short- and long-term health and behavioral risks. Studying the estimated time for a female to have her first sexual debut is important to reduce its health, demographic, and socioeconomic consequences. Thus, this study is aimed at assessing the time to first sexual experience and its determinants in Ethiopia.

**Methods:**

A survival analysis of time to first sexual experience was conducted among 6143 weighted study subjects. The data were extracted from EDHS 2016 using STATA version 16 software. A Kaplan-Meier survival curve was computed to estimate the time of first sexual experience. A log-rank test was used to compare the difference in survival curves. The Cox proportional hazard regression model was used to identify significant predictors. On multivariable analysis, variables having a *p* value of ≤ 0.05 are considered statically significant.

**Results:**

The overall median survival time was 16 years. The significant determinants of time to first sexual experience are educational level (no education (AHR = 2.72, 95% CI: 2.16, 3.39), primary education (AHR = 2.17, 95% CI: 1.79, 2.63), and secondary education (AHR = 1.47, 95% CI: 1.21, 1.77)) and wealth index (poor (AHR = 1.15, 95% CI: 1.00, 1.32)).

**Conclusion:**

About 50% of female youths have a sexual experience for the first time before their 16th birthday. The timing of the first sexual experience in Ethiopia was mainly influenced by educational level and wealth index. Universal access to education and poverty reduction should be the area of concern.

## 1. Introduction

Youth is markedly characterized by physical, emotional, and physiological changes. During this stage of life, lifelong behavioral patterns are formed. One of the changes during the youth age group is a substantial increase in sexual thoughts and feelings. Recently, early sexual experiences before the age of 15 have become more common [1]. The first sexual experience is the most significant event in a woman's life. The time it takes for a woman to have her first sexual encounter has a huge impact on her health outcome. Early-onset and negative first sexual experiences have been constructed as markers of vulnerability tied to short- and long-term health and sexual behavior risks [2, 3]. Female youths who have their first sexual experience before the age of 13 have a higher risk of contracting an STI. Following infection, the cervix becomes immature, increasing the risk of pelvic inflammatory illness, infertility, ectopic pregnancy, premature birth, and fetal abnormalities [4, 5].

Risky sexual behavior among female youths is also determined by the time of their first sexual experience. Girls who make their sexual debut before the age of 14 are less likely to utilize contraception to prevent pregnancy, are more likely to have several sex partners, experience unhappiness, poor self-esteem, and more bouts of repentance, and are more likely to contract a sexually transmitted infection [6]. Girls with low educational, economic, and cultural standing, inadequate parental supervision, parental separation, and absence of religiosity are likely to have sex at a younger age. Adolescent females who postpone sexual debut until they are 16 years old are physically and mentally healthier than those who have sexual experience at an earlier age [7].

Regarding contraceptive usage, female youths who were under 15 at their first sexual experience show a two-times-gap in contraceptive usage as compared to women who were 18 or older at their first sexual debut. Age at first sexual debut is associated with contraceptive usage later in life [8]. Early first sexual encounters increase the risk of unsafe sex, multiple relationships, and sexually transmitted infections, such as HIV/AIDS [9, 10]. Persistent gap in contraceptive usage leads to unintended pregnancy and ends with abortion [11]. Unintended pregnancy is linked to risky prenatal behaviors such as alcohol and drug abuse, as well as a poor birth outcome. It is also responsible for $11.1 billion in maternity health-care costs [12].

Indeed, recent studies have explored early sexual engagement predominantly as a possible risk factor for unfavorable social and health impacts [13]. The time at which first sexual experience is correlated with early childbearing, which is associated with a poor health outcome, consequently contributes to complications during labor and delivery as well as increases the possibility of maternal mortality and morbidity [14].

Because of Ethiopia's low economic growth, widespread poverty, and poor and insufficient health services, the repercussions of adolescent sexuality are far more serious than in developed countries. This is evident by the highest HIV prevalence. Due to early sexual debut, early marriage, sexual abuse, and violence such as rape and abduction, young Ethiopian girls are more vulnerable to HIV than boys [15]. Low educational status, ever chewing khat, region, and living in a poor community all contributed to early sexual debut among Ethiopian female youths [16].

In Ethiopia, a national adolescent and youth health strategy was formulated to address the sexual and reproductive health problems of adolescents and youth, including early sexual debut and teenage pregnancies, with the aim of increasing the median age at first sex among adolescent girls to at least 18 years [17]. However, age at first sex among adolescent girls does not show significant changes. In line with the above strategy, the results of this study are significantly important in providing relevant information in accordance with the aforementioned strategy. Even though the age of first sex among female youths has multiple health, economic, and demographic impacts, only a few related studies have been undertaken so far in Ethiopia. Most studies mainly focus on how many youths have early sexual experiences. Rather than classifying as early or not early in most studies, the current study is focused on time-to-event analysis to estimate the time for female youth to experience their first sexual encounter irrespective of what duration. Using national representative data is important in providing useful national representative information for policymakers to reduce the health, demographic, and socioeconomic consequences of the time of first sexual experience. Thus, this study is aimed at assessing the time to first sexual experience and its determinants among female youths in Ethiopia.

## 2. Methods

### 2.1. Study Setting, Data Source, Population, and Period

The Ethiopian population was estimated at 115.0 million in 2020, as per the latest census figures and projections from trading economics [18]. According to the new structure, there are eleven regions and two city administrations in the country. The administration levels went from regions to zones and through woredas. The study was conducted in Ethiopia using the 2016 Ethiopian Demographic and Health Survey data. EDHS 2016 was conducted from January 18, 2016, to June 27, 2016, based on a nationally representative sample that provides estimates at the national and regional levels as well as includes urban and rural areas. The target groups were women ages 15–49 and men ages 15–59 in randomly selected households across Ethiopia. EDHS 2016 contains detailed information on background characteristics of the respondents, fertility, marriage and sexual activity, awareness, use of family planning methods, child feeding practices, nutritional status of women and children, and adult and childhood mortality. We receive a permission letter to download EDHS 2016 data from https://www.dhsprogram.com/ after making a reasonable request. After downloading the EDHS dataset, data extraction was done to select female youth of age 15-24 years, and the weighted sample was found to be 6401. The data extraction period was from May 1 to June 1, 2022.

### 2.2. Study Variables

The outcome variable in this study was the time (age in years) at first sexual experience. The independent variables were sociodemographic factors (age, residence, religion, educational status, employment status, and household wealth index), behavioral and media exposure-related factors (alcohol drinking, cigarette smoking, chewing khat, frequency of watching television, and frequency of listening to radio).

### 2.3. Operational Definition

Age at first sexual experience: age at first intercourse (vaginal penile penetration). Sexual contacts (kissing) were not included

Event: having first sexual experience

Censored: never had sexual experience

Survival time: the time it takes to have first sexual experience (form birth to first sexual experience) in year

### 2.4. Sampling Methods

A total of 6143 weighted samples of study participants are included in this study. The EDHS 2016 sample was stratified and selected in two stages. The detailed sampling procedure is available in the EDHS 2016 report [19]. The highlighted sampling procedure for this study is indicated in Figure 1.

### 2.5. Data Processing and Analysis

STATA version 16 software was used to extract data from the EDHS 2016 individual (women) record folder. The data was coded, cleaned, and edited. Listing and sorting were done to identify any missing values. Missing values were excluded from the analysis. A Kaplan-Meier survival curve was computed to estimate the time of first sexual experience. A log-rank test was used to compare the difference in survival curves between categories of variables. Multicollinearity was checked prior to running the Cox proportional hazard regression model. The variance inflation factor result showed that the maximum VIF was 2.45 for residences and the mean VIF was 1.49. Based on the VIF result, there is no multicollinearity between covariates. Proportional hazard assumption test was checked by using the Schoenfeld residuals. In the Shenfield residual test, covariates with a *p* value of greater than 0.05 were considered to satisfy the assumption for the Cox proportional hazard regression model. Based on the global test result of the Shenfield residuals, all the covariates fulfil the PH assumption (chi − square = 14.4 and *p* value = 0.0719). Variables having a *p* value of ≤0.25 in the bivariate analysis were fitted and included in the multivariable Cox proportional hazard regression model. Both crude hazard ratio (CHR) and adjusted hazard ratio (AHR) were computed. In multivariable analysis, those variables having a *p* value of ≤0.05 are considered statistically significant.

### 2.6. Ethical Consideration

The EDHS 2016 was approved by the National Research Ethics Review Committee (NRERC) of the Ethiopian Ministry of Science and Technology. As stated in the EDHS report, participation in the study was voluntary, and verbal informed consent was also obtained [19].

## 3. Results

### 3.1. Sociodemographic Distribution of the Study Participants

6143 female youths (15–24 years) from the EDHS 2016 dataset were included to examine time to first sexual experience. Weighted frequency analysis showed that 4676 (76.11%) of respondents resided in rural areas. 2643 (43.03%) of study participants were ever married, and among those, 1018 (38.52%) were married before the age of 16 years. 2640 (42.97%) of the participants were orthodox in religion. Regarding educational status, 1230 (20.03%) of respondents have no formal education. Two thousand twenty-six (32.98%) of female youths were in the poor household wealth index category (Table 1).

### 3.2. Behavioral and Media-Related Factors of Respondents

Among the total respondents, 1972 (32.09%) and 27 (0.43%) of study participants drink alcohol and smoke cigarettes, respectively. Regarding media exposure, 1224 (18.29%) and 1086 (17.68%) of respondents watch television and listen to radio at least once a week, respectively (Table 2).

### 3.3. Sexual Debut at Different Ages

Sexual debut varied at different ages among different socioeconomic groups. The percentage of sexual debut at the age of 15 years among rural residence is 6.9%. Regarding educational status, sexual debut among those with no education at the age of 15 years is 3.1% (Table 3).

### 3.4. First Sexual Experience Status of Respondents

In this study, 2865 (46.64%) of female youth had their first sexual experience, and 3278 (53.36%) were censored (never had sex) during the follow-up time. The survival time of first sexual experience at the ages of 10, 15, and 20 years was 99.1%, 82.2%, and 10.6%, respectively. The total follow-up time contributed by all study participants was 50,719 person years. The overall median survival time was 16 years old. The median age at first marriage was 17 years.

For female youths, the minimum and maximum follow-up time to have their first sexual experience was 8 and 23, respectively (Figure 2).

The median and mean survival time quite varied among the participant characteristics. The median survival time ranges from 16 years for those with no education to 19 years for those with higher educational status. By wealth index, the median survival times for the poor, middle, and rich were 16, 16, and 17 years, respectively. The median survival time by alcohol drinking and cigarette smoking does not show a significant difference.

### 3.5. Comparisons of Survival Functions of Different Categorical Variables

The Kaplan-Meier survival curve and log-rank test were computed to compare and estimate the survivor function among different groups of variables. In the Kaplan-Meier survival curve, the lower one has a lower survival probability than the upper one—in other words, the lower curve implies a higher probability of sexual debut than the upper curve. Furthermore, the difference was described statistically by the log-rank test (Figure 3).

### 3.6. Model Selection

Model selection was done based on the baseline hazard distributional pattern. If the baseline hazard had a specific distributional pattern, a comparison will be computed by parametric survival models. If the baseline hazard has no specific distributional pattern, then the Cox proportional hazard regression model will be fitted. In this study, the baseline hazard has no distributional pattern; thus, a simple Cox regression was fitted (Figure 4).

### 3.7. Predictors of Time to First Sexual Experience

In the bivariable Cox proportional hazard regression model, residence, religion, educational status, wealth index, working status, khat chewing, frequency of watching television, and frequency of listening to radio were found to be significant at *p* value ≤0.25. In the multivariable Cox proportional hazard regression model, only educational status and wealth index were found to be predictors of time to first sexual experience.

Female youths with no formal education have more than two and half times increased hazard of first sexual experience (AHR = 2.72, 95% CI: 2.16, 3.39) than those with higher educational status. Youths with primary education had more than twofold hazard to first sexual experience (AHR = 2.17, 95% CI: 1.79, 2.63) than those with higher education. The hazard of first sexual experience among youths with secondary education was increased by 47% (AHR = 1.47, 95% CI: 1.21, 1.77) when compared to youths with higher educational status.

The hazard of first sexual experience among female youths who live in a household wealth index of poor was increased by 15% (AHR = 1.15, 95% CI: 1.00, 1.32) as compared to those who live in a rich wealth index category (Table 4).

## 4. Discussion

This study assessed time to first sexual experience and its determinants among female youths. According to the findings of this study, the median age at first sexual experience is 16 years. Level of education and wealth index were found to be predictors of time to first sexual experience.

The median age at first sexual experience is 16 years. This finding is in line with the study conducted in Nigeria (16 years) [20] and Italy (16 years) [21]. The above finding is lower than the studies done in South Africa (18.5 years) [22], Zimbabwe (18.5 years) [23], Korea (21 years) [24], China (19 years) [25], and Ireland (17 years) [26]. The possible discrepancy would be that recent advancements in technology have led to an increase in watching pornographic material, which was considered the main reason for early sexual debut [27], age differences of study population, time elapsed between studies, and behavioral variations among study participants. The median age at first sex is a general indicator of how quickly sexual activity develops among female youths. Age at first sexual debut has significant implications for youth's sexual and reproductive health thereby solidifying the need for the availability of sexual and reproductive health (SRH) educational program and service in school and community for youth, both in terms of knowledge and skill that helps youth to postpone their sexual debut.

However, the above finding is higher than the study conducted in Gambia (14 years) [28] and Brazil (14.9 years) [29]. The difference may be due to the recent decrease in early marriage in Ethiopia [30] which could be the main reason for early sexual debut [30]. Another possible reason could be an increase in youth-friendly service through time, which might have a positive impact on their knowledge of sexual issues [31].

The level of education status was a significant predictor of the time of first sexual experience. Females with no formal education have their first sexual experience more than twice as early as females with a higher educational level. Furthermore, female youths who attend primary and secondary education also have their first sexual experience at an earlier age as compared to those with higher educational attainment. This finding was supported by a study done in Gambia [28], Nekemte town [32], and North East Ethiopia [33]. The possible explanation might be that youths who are educated may have the awareness and opportunity to know the social, behavioral, and mental effects of first sexual debut. Furthermore, education may result in behavioral changes regarding alcohol consumption, cigarette smoking, and chewing tobacco, all of which are mentioned in many studies as factors for early sexual debut [33–35]. Moreover, youths who are not educated might be at risk for peer pressure which contributes to early initiation of sexual debut [36]. Thus, education may enlighten female youth about the potential impact of early sexual initiation through sex educational programs, thereby enabling them to develop a repertoire of resilience and life skills, including self-efficacy, to postpone sexual debut.

This study also found that the wealth index has a significant effect on the age at first sexual experience. Living in a household wealth index category of the poor shortens the timing of first sexual experience when compared to those in the rich category. This finding is in row with the study done in Nepal [37]. Females from low-income families may engage in earlier sexual activity in exchange for money and other benefits. Thus, poverty may have a significant impact on young people's future by leaving long-term ramifications from sexual and reproductive complications.

The strength of this study is that it uses national representative data, so it is generalizable to all Ethiopian female youths. Since the data was self-reported, it might be affected by recall bias. Because the data sources are secondary, other potential predictors of time to sexual debut are difficult to quantify. Lack of a trend analysis is also a limitation.

## 5. Conclusion

In this study, the median age at first sexual experience was 16 years. This finding is comparable with that of studies in sub-Saharan African countries. About 50% of female youths have a sexual experience for the first time before their 16th birthday. This age is the optimal age for education. Aside from the implications for her social, physical, and mental health, sexual debut at this age may result in an unintended pregnancy, preventing the female from attending school. The timing of the first sexual experience in Ethiopia was mainly influenced by the educational level and household wealth index. Increasing universal educational opportunities for Ethiopian female youth plays a paramount role in reducing the consequences of the timing of sexual debut. Policymakers should focus on the establishment of income-generating activities (entrepreneurship) and poverty reduction.

## Figures and Tables

**Figure 1:** Schematic representation of the sampling procedures in the study of time to first sexual experience and its determinants among female youths in Ethiopia, 2022. N.B: EAs = enumeration areas.

**Figure 2:** Overall Kaplan-Meier failure curve of female youth in Ethiopia, EDHS 2016.

**Figure 3:** Kaplan-Meier survival curves and log-rank tests of female youths by their characteristics in Ethiopia, EDHS 2016. N.B: KM = Kaplan-Meier.

**Figure 4:** Baseline hazard distribution plot to check whether the data has a specific distribution or not.

**Table 1:** Sociodemographic distribution of female youths (15–24 years) in Ethiopia, EDHS 2016 (*n* = 6143).

Variable	Categories	Weighted frequency	Weighted percentage	Median survival time
Age	15-19	3381	55.0%	16
	20-24	2762	44.9%	17

Residence	Urban	1467	23.9%	17
	Rural	4676	76.1%	16

Marital status	Ever married	2643	43.0%	16
	Not married	3500	56.9%	18

Age at first marriage	Less than 16	1018	38.5%	15
	16 and above	1625	61.5%	18

Religion	Orthodox	2640	42.9%	17
	Muslim	1883	30.7%	16
	Protestant	1487	24.2%	16
	Others	133	2.2%	16

Educational status of respondents	No education	1230	20.0%	16
	Primary	3333	54.3%	16
	Secondary	1184	19.3%	18
	Higher	396	6.4%	19

Wealth index	Poor	2026	32.9%	16
	Middle	1114	18.1%	16
	Rich	3003	48.8%	17

Current working status	No	4464	72.7%	16
	Yes	1679	27.3%	17

**Table 2:** Behavioral and media-related characteristic of female youths, EDHS 2016 (*n* = 6143).

Variable	Categories	Weighted frequency	Weighted percentage	Median survival time
Drinking alcohol	No	4171	67.9%	16
	Yes	1972	32.1%	17

Cigarette smoking	No	6116	99.6%	16
	Yes	27	0.4%	16

Khat chewing	No	5616	91.4%	16
	Yes	527	8.5%	16

Frequency of watching television	Not at all	4205	68.4%	16
	Less than once a week	814	13.2%	17
	At least once a week	1124	18.3%	18

Frequency of listening to radio	Not at all	3910	63.6%	16
	Less than once a week	1147	18.7%	17
	At least once a week	1086	17.7%	17

**Table 3:** Weighted frequency and percentage of sexual debut at different ages among different socioeconomic groups, EDHS 2016 (*n* = 6143).

Variable	Categories	Sexual debut at different ages		
Variable	Categories	15 years	18 years	20 years

Age	15-19	185 (3.0%)	83 (1.3%)	_____
	20-24	302 (4.9%)	343 (5.6%)	157 (2.6%)

Residence	Urban	59 (0.9%)	86 (1.4%)	59 (0.9%)
	Rural	428 (6.9%)	340 (5.5%)	98 (1.6%)

Marital status	Ever married	463 (7.5%)	389 (6.3%)	132 (2.1%)
	Not married	24 (0.4%)	37 (0.6%)	25 (0.4%)

Educational status of respondents	No education	191 (3.1%)	96 (1.6%)	18 (0.3%)
	Primary	260 (4.2%)	214 (3.5%)	77 (1.2%)
	Secondary	29 (0.5%)	83 (1.4%)	40 (0.6%)
	Higher	7 (0.1%)	32 (0.5%)	21 (0.3%)

Wealth index	Poor	989 (6.3%)	450 (2.9%)	232 (1.5%)
	Middle	329 (2.1%	270 (1.7%)	118 (0.7%)
	Rich	571 (3.6%)	571 (3.6%)	337 (2.1%)

Current working status	No	1547 (9.9%)	889 (5.7%)	399 (2.5%)
	Yes	741 (4.7%)	403 (2.6%)	287 (1.8%)

**Table 4:** Bivariable and multivariable Cox regression analysis for determinants of time to first sexual experience among female youths in Ethiopia, EDHS 2016 (*n* = 6143).

Variable	Categories	Outcome		CHR (95% CI)	AHR (95% CI)
		Censored	Event		
Residence	Urban	969	498	1	1
	Rural	2309	2366	1.59 (1.41, 1.81)	1.07 (0.91, 1.28)

Religion	Orthodox	1401	1239	1	1
	Muslim	874	1009	1.17 (1.04, 1.32)	0.93 (0.82, 1.05)
	Protestant	948	539	0.89 (0.76, 1.04)	0.86 (0.74, 1.00)
	Others	55	78	1.08 (0.89, 1.31)	0.84 (0.69, 1.02)

Educational status	No education	330	900	3.13 (2.56, 3.81)	2.72 (2.16, 3.39)^∗∗∗^
	Primary	1884	1449	2.39 (2.00, 2.85)	2.17 (1.79, 2.63)^∗∗∗^
	Secondary	824	360	1.55 (1.28, 1.88)	1.47 (1.21, 1.77)^∗∗∗^
	Higher	240	156	1	1

Wealth index	Poor	826	1200	1.52 (1.36, 1.69)	1.15 (1.00, 1.32)^∗^
	Middle	560	554	1.38 (1.21, 1.58	1.11 (0.96, 1.29)
	Rich	1893	1110	1	1

Working status	No	2369	2095	1.24 (1.11, 1.39)	1.03 (0.93, 1.16)
	Yes	909	770	1	1

Khat chewing	No	3124	2492	1	1
	Yes	154	373	1.24 (1.05, 1.46)	1.11 (0.92, 1.34)

Frequency of watching television	Not at all	2066	2139	1.57 (1.37, 1.79)	0.99 (0.84, 1.19)
	Less than once a week	480	334	1.32 (1.11, 1.57)	1.08 (0.91, 1.28)
	At least once a week	733	391	1	1

Frequency of listening to radio	Not at all	1972	1938	1.25 (1.12, 1.40)	0.99 (0.81, 1.15)
	Less than once a week	673	474	1.03 (0.89, 1.20)	1.00 (0.85, 1.18)
	At least once a week	632	454	1	1

N.B: CHR = crude hazard ratio; AHR = adjusted hazard ratio.

## Data Availability

The data for this study was obtained from the 2016 Ethiopian Demographic and Health Survey and it is available through https://www.dhsprogram.com.
